# Detecting Personal Medication Intake in Twitter via Domain Attention-Based RNN with Multi-Level Features

**DOI:** 10.1155/2022/5467262

**Published:** 2022-08-09

**Authors:** Shufeng Xiong, Vishwash Batra, Liangliang Liu, Lei Xi, Changxia Sun

**Affiliations:** ^1^Henan Agricultural University, Zhengzhou 450002, China; ^2^School of Computing and Mathematics, Keele University, Keele ST55AA, UK

## Abstract

Personal medication intake detection aims to automatically detect tweets that show clear evidence of personal medication consumption. It is a research topic that has attracted considerable attention to drug safety surveillance. This task is inevitably dependent on medical domain information, and the current main model for this task does not explicitly consider domain information. To tackle this problem, we propose a domain attention mechanism for recurrent neural networks, LSTMs, with a multi-level feature representation of Twitter data. Specifically, we utilize character-level CNN to capture morphological features at the word level. Subsequently, we feed them with word embeddings into a BiLSTM to get the hidden representation of a tweet. An attention mechanism is introduced over the hidden state of the BiLSTM to attend to special medical information. Finally, a classification is performed on the weighted hidden representation of tweets. Experiments over a publicly available benchmark dataset show that our model can exploit a domain attention mechanism to consider medical information to improve performance. For example, our approach achieves a precision score of 0.708, a recall score of 0.694, and a *F*1 score of 0.697, which is significantly outperforming multiple strong and relevant baselines.

## 1. Introduction

Social media (Twitter, Facebook, etc.) encourages users to frequently express their thoughts, opinions, and other personal information of their lives. Existing studies have demonstrated that social media messages can provide knowledge for tracking public political opinion [1], detecting news events [2], and tracking the spread of infectious diseases [3]. Some research has also shown that social media can be used as a resource for mining public health information [4–6], especially in cases where the health data from official institutions is not readily available.

In this work, we focus on the task of medication intake detection, which is an individual level surveillance of drug safety [7] in the public health domain. The goal of the task is to automatically detect tweets that express clear evidence of personal medication consumption. For example, messages like indicate the author intakes medicine while indicates no intake.

There are two types of existing methods for this emerging task in the public health domain. The first involves applying traditional classification algorithms with hand-crafted features. For example, Kiritchenko et al. [8] exploited an SVM classifier with a variety of features for this task. Another one excludes the time-consuming effort of designing hand-crafted features by using deep neural networks and directly feeding word embedding as the input. Several methods based on CNNs (Convolutional Neural Networks) have achieved good performance [9–11].

Both of them have limitations. Traditional classification methods lack nonlinear mapping ability, although they can make full use of domain knowledge information (e.g., drug lexicon and domain word clusters) [8]. The neural-based methods based on pre-trained embeddings of words [12, 13] are domain-independent and are not very effective for a specific task [14, 15], for example, our medicine intake classification task. In addition, it is not always possible to train task-specific word embeddings due to limitations on training resources. Despite some efforts to solve the problem of domain relevance at the feature level, for example, sentiment analysis on Nepali COVID-19 tweets [16], no relevant research work considering domain information has been found on our task.

To deal with the aforementioned limitations, we introduce a domain attention mechanism for recurrent neural networks with multi-level inputs to learn an informative representation of tweets. The attention mechanism enables the model the ability of learning domain-specific (medicine) matrix representation, which automatically weights the words in the text accordingly in the medication intake detection task. Meanwhile, the proposed model considers both word-level and character-level features as input features of the network. A prominent advantage of using character-level representation is that it is beneficial for many text analysis tasks [17–19], especially for informal text [20, 21], for example, tweets.

In particular, the proposed model generates word representations using a character-level CNN, which are fed to a highway network. We then concatenate them with pre-trained word embeddings, before feeding them to a BiLSTM network. Subsequently, as previously mentioned, the BiLSTM is introduced with an attention mechanism to distinctively attend on different words while learning the representation of the text. The attention-based BiLSTM also learns the representation of higher-level features in the whole text sequence of a tweet. Finally, softmax is applied to the final tweet representation for the classification task. We compared the experimental results obtained using our method with several strong and relevant baselines. We observe that our approach, with a micro-averaged F-score of 0.697 for Classes 1 and 2, achieves better performance on all other methods except ensemble approaches, which are more efficient than the standard approach. Altogether, this work introduces a novel attentional RNN framework with multi-level features that can effectively be applied to the personal medication intake detection task.

## 2. Related Work

Personal medication intake detection belongs to a short text classification task. Traditional representative methods for this task include statistical machine learning methods and deep learning methods. The vast majority of the first category is based on the vector space model, which is a typical method for tweet classification [22, 23]. Wang et al. [24] developed an SVM-based text classification algorithm. Chen et al. [25] and Jiang et al. [26] exploited the Naive Bayesian (NB) approach and KNN for this task, respectively. Wan et al. [27] implemented a new document classification method by integrating KNN and SVM, while Rogati et al. [28] investigated a large number of feature selection methods for text classification. However, these methods heavily depend on feature engineering, which cannot represent the grammatical and deep semantic information of words well.

Deep learning methods can automatically select features and therefore have become the mainstream methods for text classification in recent years. The first step is to learn word representations using related methods [29–31]. Based on them, researchers initially adopted the CNN-based method to classify texts [32, 33]. Collobert et al. [33] extracted local features by using a convolutional layer. Kim [34] constructed a single-layer convolution network for sentence classification. Kalchbrenner et al. [35] proposed a CNN model with multi-layer dynamic k-Max pooling, taking random low-dimensional word vectors as input. Er et al. [36] developed an attention-based pooling component, which has the ability to obtain more semantic information. Yin et al. [37] developed a multi-channel variable-size CNN, which can support multiple pre-trained word embeddings and variable-size convolution kernel to obtain multi-granularity phrase features. Recently, the RNN-based model shows good performance. Lee et al. [38] exploited a convolutional recurrent neural network to process long text sequences. Lai et al. [39] proposed a bi-directional recurrent structure that can utilize the context information of words to classify text.

In addition, the participating systems of the SMM4H shared task are related to our method. These systems can be also divided into traditional statistic methods [8, 40] and neural network methods [10, 41]. Due to the characteristics of pursuing high-performance scores in evaluation tasks, most of them used ensemble technology. More details can be referred to the literature [9].

## 3. Background

### 3.1. Personal Medication Intake Detection

The primary objective of the personal medication intake detection task is the automatic classification of tweets mentioning medication intake, which is an emerging research topic in the public health domain based on social media. This is a three-class text classification task. Each medicine-mentioned tweet needs to be grouped into one of three categories: definite intake, non-intake, and possible intake. The details of these categories are as follows.

- Define intake (Class 1)-The user expresses clear evidence of personal medication consumption, for example, “Benadryl and Tylenol are the only things saving me at night these last few nights.”
- Possible intake (Class 2)-It is suggested that one poster may have taken the medication, but there is no clear evidence, for example, “I would love to intravenously pump Motrin and caffeine into my body immediately.”
- Non-intake (Class 3)-There is no evidence showing that the user has consumed the medication, while it only mentions medication names, for example, “stay out of the heat, only drink water, and stay off your feet for a day or two. Tylenol is all you can take for pain.”

### 3.2. Character Convolutional Neural Network (CNN)

Character Convolutional Neural Network (C-CNN) [17, 42] is fed characters instead of words, as in traditional CNN. Given an input word *w*, which can be seen as a character sequence *C*={*c*_1_, *c*_2_,…, *c*_*n*_}, where *n* is the length of the word. The C-CNN applies the convolution operation on the character sequence to generate the feature map *V*_1_ as follows:

(1) $$\begin{array}{c} V_{1}=\text{Conv}\left(W,C\right)+b, \end{array}$$

where Conv denotes the convolution kernel and *W* and *b* are learnable parameters. In practice, there are different convolution kernels for catching various features. A pooling layer, which is utilized to compress and obtain crucial features for the next layer, is usually applied after the convolution layer. The computing process can be written as

(2) $$\begin{array}{c} V_{2}=\text{Pooling}\left(V_{1}\right). \end{array}$$

There are two common pooling operations: max pooling and mean pooling. For example, max pooling chooses the maximum value in a pooling window as the output result of the pooling process. Several combinations of convolution and pooling layers could be used in practice for specific tasks.

### 3.3. Bi-Directional Long Short Term Memory (BiLSTM)

The Long Short Term Memory (LSTM) network was introduced by Hochreiter et al. [43] and was refined and promoted by many works [44–46]. The LSTM solves the long-term dependency problem in the RNN model [47]. Given a sequence *X*={*x*_1_, *x*_2_,…, *x*_*n*_} as input, the operations performed by the LSTM units are as follows:

(3) $$\begin{array}{c} s_{t}=\left[h_{t-1},x_{t}\right],\\ f_{t}=W_{f}\cdot s_{t}+b_{f},\\ i_{t}=W_{i}\cdot s_{t}+b_{i},\\ u_{t}=W_{u}\cdot s_{t}+b_{u},\\ C_{t}=\delta \left(f_{t}\right)*C_{t-1}+\delta \left(i_{t}\right)*\text{tan}h\left(u_{t}\right),\\ o_{t}=W_{o}\cdot \left(s_{t}+b_{o}\right),\\ h_{t}=\delta \left(o_{t}\right)*\;\tan h\left(C_{t}\right), \end{array}$$

where *h*_*t*_ is the output of the LSTM at time step *t*. *W* and *b* are the weights and bias, respectively, and *δ* is a sigmoid layer. In many NLP tasks, a bi-directional LSTM is used to obtain forward and backward information of words in a sequence. In BiLSTMs, it concatenates the outputs of the forward and backward hidden states as its output:

(4) $$\begin{array}{c} h_{t}=\left[\overset{⟶}{h_{t}},\overset{\leftarrow }{h_{t}}\right]. \end{array}$$

## 4. Methods

Our proposed model combines the C-CNN and BiLSTM. It also introduces an attention mechanism in the BiLSTM for the personal medication intake detection task. The model consists of a character-level word embedding component, a word-level feature representation component (Character Language Model, CLM) that uses C-CNN, a sentence-level feature representation component using BiLSTM, and a Domain Attention Component (DAC). An overview of our model is shown in Figure 1.

Since tweets are mostly informal, traditional word embeddings cannot represent it well. Therefore, we use a Character Language Model (CLM) to capture morphological features at the word level. Firstly, a character embedding *e*_*c*_ is created for each character in a word. Our model then converts the character embedding sequence into a vector using a CLM, which is a kind of C-CNN network. The structure of the CLM is as shown on the right in Figure 1.

Specifically, for every word *w* in a sentence, after passing it to convolutional and max pooling layers, our model utilizes a highway network[42, 48] to regulate the information flow:

(5) $$\begin{array}{c} \hat{C}=g\left(W_{h}\cdot V_{2}+b_{h}\right)\cdot t+V_{2}\cdot \left(1-t\right),\\ t=H\left(W_{t}\cdot V_{2}+b_{t}\right), \end{array}$$

where *H* is a nonlinear function, *V*_2_ is calculated by equation (2), and *t* and (1 − *t*) are called the transform gate and carry gate, respectively.

After obtaining ${\hat{C}}_{i}$, the representation of the *i*-th word at character-level, we concatenate it with its word embedding *e*_*i*_ to generate the final representation of the word:

(6) $$\begin{array}{c} {\hat{e}}_{i}=\left[\hat{C},e_{i}\right]. \end{array}$$

Subsequently, we feed a sentence $s=\left({\hat{e}}_{1},{\hat{e}}_{2},{\hat{e}}_{3},\ldots {\hat{e}}_{n}\right)$ into a BiLSTM network to get the hidden states *h*=(*h*_1_, *h*_2_, *h*_3_,…, *h*_*n*_). In our experiments, we treat each tweet as one sentence and yet achieve good results since most of the tweets in our dataset are too short and mostly contain one or two sentences.

At this stage, the model performs a general processing on tweets. Therefore, for the medicine intake detection task, we introduce a DAC to attend to the specific domain information that is being used to detect a specific condition. The DAC aims to weigh the informative words for medicine intake highly. First, the result $\hat{h_{k}}$ obtained by inputting *h*_*k*_ into a single-layer perceptron is used as the hidden representation of *h*. The weight value of a word is determined by the similarity of $\hat{h_{k}}$ and a parameter *D*, here *D* can be seen as a domain context vector. After processing using a softmax function, a normalized attention weight matrix is obtained, which indicates the weight of each word in a sentence. Finally, the tweet representation *u* can be calculated as the weighted summation of the words in it. The output is computed as follows:

(7) $$\begin{array}{c} {\hat{h}}_{k}=\text{tan}h\left(W_{a}\cdot \left(h_{k}+b_{a}\right)\right),\\ a_{k}=\frac{\exp\left({\hat{h}}_{k}^{⊤}\cdot D\right)}{\Sigma_{k}\left({\hat{h}}_{k}^{⊤}\cdot D\right)},\\ u=\sum_{k}a_{k}\cdot {\hat{h}}_{k}, \end{array}$$

where *W*_*a*_ and *b*_*a*_ are the weight and bias, respectively. *a*_*k*_ stands for the attention value of the *k*-th word and measures the weight of each word in the sentence.

The vector representing the whole text sequence from a tweet or the tweet vector *u* is a higher-level representation and can be used directly as a feature for medicine intake detection:

(8) $$\begin{array}{c} p=\text{softmax}\left(W_{s}\cdot \left(u+b_{s}\right)\right). \end{array}$$

The final optimization objective is to minimize the negative log likelihood of the correct labels:

(9) $$\begin{array}{c} L=-\sum_{d}\hat{p}\text{log}p, \end{array}$$

where $\hat{p}$ represents the ground-truth label of the tweet.

## 5. Experiments

### 5.1. Dataset

Our experiments were conducted on a publicly available dataset from the 2nd SMM4H (Social Media Mining for Health) Shared Task on the AMMIA 2017 website. Using the Twitter download script and the tweet dataset description file provided by the organizers, we did not collect all the tweets since some of them are not available.  Table 1 summarizes the statistics for the dataset. Classes 1, 2, and 3 stand for personal medication intake, possible medication intake, and no medication intake, respectively. Our training dataset is a combination of the originally provided training and validation datasets. We utilize 10-fold cross-validation when training our model.

### 5.2. Model Configuration and Training

We use pre-trained word embeddings to initialize the input of the neural network model. This is highly useful for NLP tasks [49, 50]. In our work, we use the embeddings trained by a word2vec model on Twitter data [51], which are of 400 dimensions. For character embeddings, we use a random initialization since there are no publicly available character embeddings in this case.

Within our experiments, we have two types of parameters, hyper-parameters and other settings. Specifically, the character embedding dimension is 15, the dimension of the hidden layer is 300, and the CLM has filters of width [1, 2, 3, 4] of size [15, 30, 45, 60] for a total of 180 filters. Additionally, the batch size, the learning rate, the dropout rate, and the *L*2 normalization factor are set to 100, 3*e* − 4, 0.3, and 5*e* − 7, respectively. In our training process, we used early stopping with a patience value of 40.

### 5.3. Baselines

We conducted comparative studies involving experiments with several baseline methods on the dataset, including neural network methods, traditional machine learning algorithms, and state-of-the-art methods for this task. In the first category, we choose the NB and SVM algorithms:

  NB is a Naive Bayes classifier in which *n*-grams (*n* = 1, 2, 3) are used as features.
  SVM is a Support Vector Machine classifier with *n*-grams (*n* = 1, 2, 3) features.
  The neural network model is currently the dominant method for text processing. We chose the following representative methods:
  BiLSTM uses a traditional bi-directional LSTM model for medicine intake detection, which represents a sentence with the hidden state of the last word of it.
  CharCNN [18] is a classical model which performs text classification by using a character-level convolutional network.
  AttRNN [52] concatenates the last hidden state, the first hidden states of an RNN with an attentive representation of a hidden state sequence as the features of a text sequence.
  The third group is the top three systems from the SMM4H Shared Task:
  InfyNLP [10] is the first system in the 2nd SMM4H Shared Task at AMIA 2017. It uses a stacked ensemble of shallow CNNs modeled as a classifier for this task.
  UKNLP [41] is the second system in the Shared Task which utilizes a CNN network with a self-attention component.
  NRC-Canada [8] exploited the SVM classifier with a variety of hand-crafted features, which is the third system on the SMM4H Shared Task.

### 5.4. Results and Discussion

Table 2 presents the performance of the different methods. We presented the micro-averaged Precision, Recall, and *F*1 scores of Class 1 (personal medication intake) and Class 2 (possible medication intake). The best results are shown in bold text. The results with “^#^” are copied from their original papers. Following the setting in the SMM4H shared task, we report the micro-averaged scores over Class 1 and Class 2. It was observed that the proposed model performs the best over the *F*1 score against strong baselines and top systems in the SMM4H shared task. Compared with other neural classification methods, the proposed domain attention component and CLM in our model improve the performance in the context of the task at hand. CharCNN and AttRNN methods perform less than our method, while BiLSTM performs poorly in this group because they are proposed for general text classification tasks, for example, topic classification. The former two methods perform better than BiLSTM because they introduce character-level information and attention components. NB and SVM, as they are represented in traditional machine methods, perform poorly because they cannot fully capture text semantic information compared to the NN model. At the performance of the top three systems is not as good as our method.

### 5.5. Ablation Test

In this subsection, we discuss the impact and contribution of the different components of our model. Specifically, we tested 3 settings. The first, we dismissed CLM only. In this case, the model did not capture character-level features. In the next setting, we remove the DAC only. Similarly, the model did not care about the domain information. Finally, we dismiss both CLM and DAC. In this case, the model degenerates to BiLSTM, which only just uses word-level features via BiLSTM encoding.  Table 3 reports the results of this ablation study.

It is clear that both CLM and DAC are critical to the performance of our model. Removing one or both of them can cause performance degradation. In particular, we also observe that CLM seems to be less important than DAC, which means that the performance drops more as compared to removing CLM.

## 6. Conclusion and Future Works

Personal medication intake detection, aiming to automatically detect tweets that express clear evidence of personal medication consumption, is an essential research topic in the surveillance of drug safety. In this work, we proposed a domain attention component for recurrent neural networks, for example, LSTM, with multi-level feature representation of text from Twitter. Through experiments on the public benchmark dataset, we validated the performance of our model. Our model obtains the best performance of 0.697 *F*1 score. Compared with multiple strong baselines, it showed a significant performance improvement.

Our method still has limitations on domain-specific knowledge representation due to the representation ability of the neural network model itself. Thus, it would be interesting to combine the knowledge base, for example, Knowledge Graph, with our model to obtain richer domain information for this task.

## Figures and Tables

**Figure 1:** Framework of our model.

**Table 1:** Statistics of the dataset.

	Class 1	Class 2	Class 3	Total
Train	1648	2650	4246	8544
Test	1444	2267	2593	6304

**Table 2:** Comparison results.

Model	Precision	Recall	*F*1
NB	0.675	0.631	0.650
SVM	0.679	0.664	0.668
BiLSTM	0.683	0.672	0.678
CharCNN	0.681	0.697	0.689
AttRNN	0.704	0.677	0.688
InfyNLP	0.725^#^	0.664^#^	0.693^#^
UKNLP	0.701^#^	0.677^#^	0.689^#^
NRC-Canada	0.704^#^	0.635^#^	0.668^#^
Our model	0.708	0.694	0.697

**Table 3:** Comparison results with different settings.

Model	Precision	Recall	*F*1
w/o CLM and DAC	0.683	0.672	0.678
w/o CLM	0.701	0.683	0.693
w/o DAC	0.669	0.713	0.691
Full model	0.708	0.694	0.697

## Data Availability

The data used to support the findings of this study have been deposited in the website https://healthlanguageprocessing.org/sharedtask2/smm4h-sharedtask-2017/

## References

[1] O’Connor B., Balasubramanyan R., Routledge B. R., Smith N. A. From tweets to polls: linking text sentiment to public opinion time series.

[2] Popescu A.-M., Pennacchiotti M. Detecting controversial events from twitter.

[3] Lamb A., Paul M. J., Dredze M. Separating fact from fear: tracking flu infections on twitter.

[4] Liu L., Kunyan W., Xingting Z., Weng D., Gao L., Lei J. (2018). The current status and a new approach for Chinese doctors to obtain medical knowledge using social media: a study of WeChat. *Wireless Communications and Mobile Computing*.

[5] Sinnenberg L., Buttenheim A. M., Padrez K., Mancheno C., Ungar L., Merchant R. M. (2017). Twitter as a tool for health research: a systematic review. *American Journal of Public Health*.

[6] Freifeld C. C., Brownstein J. S., Menone C. M. (2014). Digital drug safety surveillance: monitoring pharmaceutical products in twitter. *Drug Safety*.

[7] Klein A., Sarker A., Rouhizadeh M., O’Connor K., Gonzalez G. (2017). Detecting personal medication intake in twitter: an annotated corpus and baseline classification system. *BioNLP 2017*.

[8] Kiritchenko S., Mohammad S. M., Morin J., de Bruijn B. NRC-Canada at SMM4H shared task: classifying tweets mentioning adverse drug reactions and medication intake.

[9] Sarker A., Belousov M., Friedrichs J. (2018). Data and systems for medication-related text classification and concept normalization from Twitter: insights from the Social Media Mining for Health (SMM4H)-2017 shared task. *Journal of the American Medical Informatics Association*.

[10] Friedrichs J., Mahata D., Gupta S. InfyNLP at SMM4H task 2:stacked ensemble of shallow convolutional neural networks for identifying personal medication intake from twitter.

[11] Mahata D., Friedrichs J., Shah R. R., Jiang J. (2018). Detecting personal intake of medicine from twitter. *IEEE Intelligent Systems*.

[12] Schwenk H. (2007). Continuous space language models. *Computer Speech & Language*.

[13] Bengio Y., Courville A., Vincent P. (2013). Representation learning: a review and new perspectives. *IEEE Transactions on Pattern Analysis and Machine Intelligence*.

[14] Fu P., Lin Z., Yuan F., Wang W., Meng D. Learning sentiment-specific word embedding via global sentiment representation.

[15] Zamani H., Croft W. B. Relevance-based word embedding.

[16] Ren Y., Wang R., Ji D. (nov 2016). A topic-enhanced word embedding for Twitter sentiment classification. *Information Sciences*.

[17] Dos Santos C. N., Zadrozny B. Learning character-level representations for part-of-speech tagging.

[18] Zhang X., Zhao J., LeCun Y., Cortes C., Lawrence N. D., Lee D. D., Sugiyama M., Garnett R. (2015). Character-level convolutional net-works for text classification. *Advances in Neural Information Processing Systems 28*.

[19] Kavuluru R., Rios A., Tran T. Extracting drug-drug interactions with word and character-level recurrent neural networks.

[20] Vosoughi S., Vijayaraghavan P., Roy D. Tweet2Vec: learning tweet embeddings using character-level CNN-LSTM encoder-decoder.

[21] Liang D., Xu W., Zhao Y. Combining word-level and character-level representations for relation classification of informal text.

[22] Sitaula C., Basnet A., Mainali A., Shahi T. B. (2021). Deep learning-based methods for sentiment analysis on Nepali COVID-19-related tweets. *Computational Intelligence and Neuroscience*.

[23] Shahi T. B., Sitaula C., Paudel N. (2022). A hybrid feature extraction method for Nepali COVID-19-related tweets classification. *Computational Intelligence and Neuroscience*.

[24] Wang Z. Q., Sun X., Zhang D. X., Li X. An optimal SVM-based text classification algorithm.

[25] Chen J., Huang H., Tian S., Qu Y. (2009). Feature selection for text classification with Naïve Bayes. *Expert Systems with Applications*.

[26] Jiang S., Pang G., Wu M., Kuang L. (2012). An improved K-nearest-neighbor algorithm for text categorization. *Expert Systems with Applications*.

[27] Wan C. H., Lee L. H., Rajkumar R., Isa D. (2012). A hybrid text classification approach with low dependency on parameter by integrating K-nearest neighbor and support vector machine. *Expert Systems with Applications*.

[28] Rogati M., Yang Y. High-performing feature selection for text classification.

[29] Bengio Y., Ducharme R., Vincent P., Jauvin C. (2003). A neural probabilistic language model. *Journal of Machine Learning Research*.

[30] Pennington J., Socher R., Manning C. Glove: global vectors for word representation.

[31] Mikolov T., Sutskever I., Chen K., Corrado G. S., Dean J. Distributed representations of words and phrases and their compositionality.

[32] Sitaula C., Shahi T. B. (2021). Multi-channel CNN to classify Nepali covid-19 related tweets. https://arxiv.org/.

[33] Collobert R., Weston J., Bottou L. E. O., Karlen M., Kavukcuoglu K., Kuksa P. (2011). Natural language processing (almost) from scratch. *Journal of Machine Learning Research*.

[34] Kim Y. Convolutional neural networks for sentence classification.

[35] Kalchbrenner N., Grefenstette E., Blunsom P. A convolutional neural network for modelling sentences.

[36] Er M. J., Zhang Y., Wang N., Pratama M. (2016). Attention pooling-based convolutional neural network for sentence modelling. *Information Sciences*.

[37] Yin W., Schütze H. Multichannel variable-size convolution for sentence classification.

[38] Lee J. Y., Dernoncourt F. Sequential short-text classification with recurrent and convolutional neural networks.

[39] Lai S., Xu L., Liu K., Zhao J. Recurrent convolutional neuralnet works for text classification.

[40] Hb B. G., Kp S. NLP_CEN_AMRITA @ SMM4H:health care text classification through class embeddings.

[41] Han S., Tran T., Rios A., Kavuluru R. Team UKNLP: detecting ADRs, classifying medication intake messages, and normalizing ADR mentions on twitter.

[42] Kim Y., Jernite Y., Sontag D., Rush A. M. Character-aware neural language models.

[43] Hochreiter S., Schmidhuber J. (1997). Long short-term memory. *Neural Computation*.

[44] Graves A., Fernández S., Schmidhuber J. Bidirectional LSTM net-works for improved phoneme classification and recognition.

[45] Gers F. A., Schmidhuber J., Cummins F. A. (2000). Learning to forget:continual prediction with LSTM. *Neural Computation*.

[46] Sundermeyer M., Schlüter R., Ney H. LSTM neural networks for language modeling.

[47] Pearlmutter B. A. (1989). Learning state space trajectories in recurrent neural networks. *Neural Computation*.

[48] Srivastava R. K., Greff K., Schmidhuber J., Cortes C., Lawrence N. D., Lee D. D., Sugiyama M., Garnett R. (2015). Training very deep networks. *Advances in Neural Information Processing Systems 28*.

[49] Qi Y., Sachan D., Felix M., Padmanabhan S., Neubig G. When and why are pre-trained word embeddings useful for neural machine translation?.

[50] Xu H., Liu B., Shu L., Yu P. S. Double Embeddings and CNN-Based Sequence Labeling for Aspect Extraction.

[51] Godin F., Vandersmissen B., De Neve W., De Walle R. MultimediaLab @ ACL WNUT NER shared task: named entity recognition for twitter microposts using distributed word representations.

[52] Du C., Huang L. (2018). Text classification research with attention-based recurrent neural networks. *International Journal of Computers, Communications & Control*.

